# QKI5-mediated alternative splicing of the histone variant macroH2A1 regulates gastric carcinogenesis

**DOI:** 10.18632/oncotarget.8739

**Published:** 2016-04-15

**Authors:** Feng Li, Ping Yi, Jingnan Pi, Lanfang Li, Jingyi Hui, Fang Wang, Aihua Liang, Jia Yu

**Affiliations:** ^1^ Institute of Biotechnology, Key Laboratory of Chemical Biology and Molecular Engineering of National Ministry of Education, Shanxi University, Taiyuan, PR China; ^2^ Department of Biochemistry, Institute of Basic Medical Sciences, Chinese Academy of Medical Sciences (CAMS) & Peking Union Medical College (PUMC), Beijing, PR China; ^3^ Department of Obstetrics and Gynecology, Research Institute of Surgery, Daping Hospital, Third Military Medical University, Chongqing, PR China; ^4^ State Key Laboratory of Molecular Biology, Shanghai Institutes for Biological Sciences, Chinese Academy of Sciences, Shanghai, PR China

**Keywords:** QKI5, macroH2A1, alternative splicing, CCNL1, gastric cancer

## Abstract

Alternative pre-mRNA splicing is a key mechanism for increasing proteomic diversity and modulating gene expression. Emerging evidence indicated that the splicing program is frequently dysregulated during tumorigenesis. Cancer cells produce protein isoforms that can promote growth and survival. The RNA-binding protein QKI5 is a critical regulator of alternative splicing in expanding lists of primary human tumors and tumor cell lines. However, its biological role and regulatory mechanism are poorly defined in gastric cancer (GC) development and progression. In this study, we demonstrated that the downregulation of QKI5 was associated with pTNM stage and pM state of GC patients. Re-introduction of QKI5 could inhibit GC cell proliferation, migration, and invasion *in vitro* and *in vivo*, which might be due to the altered splicing pattern of macroH2A1 pre-mRNA, leading to the accumulation of macroH2A1.1 isoform. Furthermore, QKI5 could inhibit cyclin L1 expression via promoting macroH2A1.1 production. Thus, this study identified a novel regulatory axis involved in gastric tumorigenesis and provided a new strategy for GC therapy.

## INTRODUCTION

Alternative splicing generates multiple different mRNAs and downstream proteins from a single gene through the inclusion or exclusion of specific exons [1, 2]. This process occurs in 95% of all multi-exonic genes, and dysregulation of splicing underlies many human diseases, including cancer. Recently, the large-scale transcriptome analysis has indicated the existence of cancer-specific splicing patterns [3–5]. The ability to commandeer alternative splicing is beneficial to cancer cells if early developmental stage isoforms critical for proliferation or apoptosis are expressed. For example, BCL2L1 possesses an alternative 5′ splice site after exon 2, which can produce long (BCL-X_L_) and short (BCL-X_S_) isoform proteins [6]. BCL-X_S_ promotes apoptosis, whereas BCL-X_L_, which shows a predominant expression in multiple cancers, exhibits anti-apoptotic effects [7]. Metabolic pathways are also frequently altered in cancer, as the Warburg effect, a shift from oxidative phosphorylation to aerobic glycolysis, is partly driven by alternative splicing of the pyruvate kinase M (PKM) gene [8]. In the alternative splicing of PKM mRNA, exons 9 and 10 are mutually exclusive, resulting in the adult isoform PKM1 (exon 9) or the tumor isoform PKM2 (exon 10). PKM2 is widely expressed in cancer cells, and replacement of PKM2 with PKM1 reverses the Warburg effect and increases oxidative phosphorylation [9, 10]. In summary, during carcinogenesis, aberrant splicing of oncogenes can produce constitutively active variants that confer new survival or proliferative abilities. By contrast, a tumor suppressor with aberrant splicing can result in an altered reading frame or a premature stop codon, which will decrease the total protein level or its tumor-suppressive capacity.

H2A, together with H2B, H3, and H4, organizes the canonical nucleosome architecture of eukaryotic genomes and is locally modified in a multitude of ways for various regulatory purposes [11, 12]. A group of H2A-type histone variants (macroH2A1.1, macroH2A1.2, and macroH2A2), collectively referred to as macroH2As, contain an amino-terminal histone-like region and a carboxyl-terminal 30 kDa globular “macrodomain” [13]. MacroH2A1 is one such histone variant that can substitute for at least one copy of H2A in a subset of nucleosomes in vertebrates. MacroH2A1 can be produced as one of two alternatively spliced mRNAs, either macroH2A1.1 or macroH2A1.2. The macrodomain of macroH2A1.1 can interact with NAD^+^-derived small molecules, whereas macroH2A1.2's macrodomain cannot [14–16]. Current data from several groups have demonstrated that macroH2A1 plays important roles in both tumor suppression and differentiation, and the alteration in macroH2A1 splicing and expression occurs in a variety of cancers, including testicular, lung, urinary bladder, cervical, breast, colon, ovarian, and endometrial cancers [16–18]. However, the involvement of macroH2A1 splicing in gastric cancer (GC), the factors regulating the splicing of macroH2A1, and the biological role of macroH2A1 splicing are largely unknown in gastric carcinogenesis.

Multiple RNA-binding proteins function as splicing regulators to interact with spliceosomes or other splicing regulators. The role of splicing regulators in cancer is best demonstrated by the RNA-binding protein, SRSF1, which functions as an oncogene to regulate alternative splicing of genes involved in cell growth and apoptosis [19–22]. Many other RNA-binding proteins also exhibit changed expression in tumor tissues, but their functions and targets during cancer development remain elusive. In this study, we demonstrated that the expression of the splicing factor Quaking (QKI) was significantly downregulated in GC and its downregulation was associated with metastasis, tumor stage, and shortened survival of GC patients. Furthermore, we showed that QKI inhibited GC cell proliferation, migration, and invasion at least in part through regulating the alternative splicing of macroH2A1. The reduced expression of the alternatively spliced form macroH2A1.1 was due to the downregulation of QKI, which could enhance the splicing of macroH2A1.1 in GC cells. Additionally, cyclin L1 (CCNL1) was validated as a downstream target of macroH2A1.1, and it was important for tumor suppressor activity in GC. Our study established the critical role of the QKI-mH2A1.1-CCNL1 axis in GC development, and targeting this pathway offers a promising strategy for GC therapy.

## RESULTS

### Aberrant expression of QKI in human GC tissues and cell lines

To determine the expression of splicing factor QKI (including QKI5, QKI6, and QKI7) in GC, quantitative PCR(qPCR) analysis was conducted in 100 pairs of clinic GC tissue and matched adjacent normal tissue samples. Among them, 84 cases (84%) showed reduced levels of QKI mRNA in tumor tissues compared with their normal tissues, whereas only 16 cases (16%) showed upregulated QKI mRNA level in GC (Figure 1A). Therefore, QKI was significantly downregulated in GC tissues compared with adjacent normal tissues (Figure 1A, p < 0.001, GC vs. normal). To further study the relationship between QKI level and clinicopathological factors of GC, the relative level of QKI in GC tissues was statistically analyzed (non-parametric test). Interestingly, we found that a low QKI level was associated with GC pM stage (Figure 1B, p < 0.001, metastasis vs. non-metastasis) and pTNM stage (Figure 1C, p = 0.01, stage I vs. II; p = 0.01, stage III vs. IV) in GC patients. However, no significant difference was found between the expression of QKI mRNA and other clinicopathologic characteristics, including gender, age, position, Borrmann typing, venous invasion, pT stage and pN stage in GC (data not shown). Additionally, GC patients with low QKI expression had markedly worse overall and disease-free survival compared with those with high QKI expression (Figure 1D and Supplementary Table 2).

**Figure 1:** Expression of QKI in GC tissues and cell lines **A.** QKI mRNA level was detected in 100 pairs of GC tissues and adjacent normal regions by RT-qPCR. **B.** The Statistical analysis of the association between QKI level and pM stage (no metastasis and metastasis); **C.** Statistical analysis of the association between QKI level and pTNM stage (I, II, III and IV); **D.** Immunoblotting analysis of QKI proteins in 10 pairs of GC samples. GAPDH was used as a loading control. The QKI5 expression level was normalized to loading control and shown in the histogram. (n = 10). **E.** Statistical analysis of survival probability of QKI high- (n = 11) and low-expressing (n = 52) GC patients using Kaplan–Meier analysis. Statistical analysis is described in the Materials and Methods. **F.** Level of QKI5 protein in GC cell lines (AGS, MKN-45, SGC-7901, BGC-823, HGC-27, and MGC-803) relative to two normal control samples; For all qPCR results, the data are presented as the mean ± SEM, and the error bars represent the standard deviation obtained from three independent experiments. * *p* < 0.05; ** *p* < 0.01.

To further validate the above results, we examined the protein levels of QKI in 10 pairs of clinic GC samples and their controls. In parallel with mRNA expression alterations, the protein level of QKI5, the dominant isoform in GC cells, among eight out of 10 paired GC samples were significantly reduced (> 1.6-fold) in tumor tissues compared with that in adjacent normal tissues (Figure 1E). Moreover, we used two normal GC samples and six GC cell lines (BGC-823, AGS, MKN-45, SGC-7901, HGC-27, and MGC-803) to analyze the QKI5 protein level. The results showed that QKI5 was markedly reduced in GC cell lines in comparison with normal controls (Figure 1F). These results indicated that the dysregulation of QKI in GC patients might suggest a potential tumor suppressor role of QKI in GC tumorigenesis.

### QKI5 inhibits GC cell proliferation, migration, and invasion

The downregulated QKI5 expression in GC samples prompted us to explore the possible roles of QKI5 in GC tumorigenesis. To assess the role of QKI5 in the pathogenesis of GC, we selected two cell lines HGC-27 and MGC-803, in which the expression level of QKI5 was relatively lower than others (Figure 1F). A construct containing QKI5 ORF (pcDNA-QKI5) was transfected into HGC-27 and MGC-803 cells, and the efficiency of QKI5 overexpression was subsequently confirmed by immunoblotting (Figure 2A). The intracellular level of QKI5 protein was enhanced by 3.9 and 3.6-fold in HGC-27 and MGC-803 cells treated with pcDNA-QKI5 than the empty vector pcDNA, respectively (Figure 2A). Accordingly, ectopic expression of QKI5 showed a significantly slower proliferation rate than control cells as determined by CCK-8 assay (Figure 2B). Furthermore, we examined the effects of QKI5 on the apoptosis of HGC-27 and MGC-803 cells receiving QKI5 or not via flow cytometry. The results showed that QKI5 overexpression increased both the early and late apoptosis of HGC-27 and MGC-803 cells compared with the control group (Figure 2C).

**Figure 2:** Functional analysis of QKI5 in GC cells **A.** QKI5 levels were detected in HGC-27 and MGC-803 cells after treatment with pcDNA-QKI5 or pcDNA empty vector by immunoblotting; **B.** Cell proliferation assay of HGC-27 and MGC-803 cells after treatment with pcDNA-QKI5 or pcDNA using CCK-8; **C.** Flow cytometry was conducted to examine the apoptosis of HGC-27 and MGC-803 cells after treatment with pcDNA-QKI5 or pcDNA and staining with apoptosis markers (FITC-Annexin V and PI). In the apoptosis map, FITC-Annexin V+/PI+ indicates late apoptosis, FITC-Annexin V+/PI− indicates early apoptosis, and FITC-Annexin V−/PI− indicates normal live cells. **D.** Wound healing assays of HGC-27 and MGC-803 cells after treatment with pcDNA-QKI5 or pcDNA. The relative ratio of wound closure per field is shown in the right; **E.** Transwell analysis of HGC-27 and MGC-803 cells after treatment with pcDNA-QKI5 or pcDNA. The relative ratio of invasive cells per field is shown in the right. For all qPCR results, the data are presented as the mean ± SEM, and the error bars represent the standard deviation obtained from three independent experiments. * *p* < 0.05; ** *p* < 0.01.

Based on the correlation between QKI5 level and GC metastasis, we proposed that this splicing factor might correlate with regulating cell migration and invasion of GC cells. To test this hypothesis, cell migration and invasion assays were performed in HGC-27 and MGC-803 cells transfected with pcDNA-QKI5 or empty pCDNA. As a result, wound healing assay showed that cell migration was reduced in QKI5-overexpressed GC cells compared with the controls (Figure 2D). Moreover, transwell invasion assay indicated a significant reduction in cell invasiveness after pcDNA-QKI5 transfection into both HGC-27 and MGC-803 cells (Figure 2E). All these results suggested that QKI5 may act as a tumor suppressor by inhibiting cell proliferation, migration and invasion, as well as promoting cell apoptosis, in GC cells.

### QKI5 inbibits tumor cell growth and metastasis *in vivo*

To further verify the findings *in vitro*, an *in vivo* mouse model was also included. MGC-803 cells infected with lentivirus carrying QKI5 ORF (QKI5) or not (control) were resuspended in PBS and injected subcutaneously (s.c.) into the posterior flank of nude mice. The animals were sacrificed after seven weeks. QKI5 overexpression resulted in significantly slower tumor growth (Figure 3A and 3B), with a mean final tumor volume of 92.4 mm^3^, compared with 587 mm^3^ in the control group (Figure 3C). Immunohistochemistry was performed to detect the expression of Ki-67 and caspase-3 in randomly selected tumors derived from QKI5- or control-transduced MGC-803 cells. As a result, the QKI5-injected tumors expressed lower levels of Ki-67 but higher levels of caspase-3, further indicating retarded GC cell growth (Figure 3D).

**Figure 3:** QKI5 suppresses GC cell growth and metastasis *in vivo* **A.** Xenograft model in nude mice. QKI5-and control-transfected MGC-803 cells were injected s.c. into the posterior flank of nude mice. The graph is representative of tumors in mice at seven weeks after inoculation. **B.** The graph is representative of excised tumors from killed mice. **C.** Tumor volume was calculated and all data are shown as the mean ± SD. **D.** Pathology analysis of tumor sections from xenograft mice. H&E staining and labeling with anti-Ki-67 and anti-caspase3 was performed. Bars: 20 μm. **E.** Nude mice were injected with MGC-803 cells infected with QKI5 or control lentivirus through the lateral tail vein. Five weeks after the injection, the mice were sacrificed, and the lungs and livers were dissected for microscopic histology. **F.** Histological analysis of sections from livers (the upper panel) and lungs (the lower panel) of mice as described in E. **G.** Quantification of visible liver (the left panel) and lung (the right panel) metastases counted using a microscope.

We further conducted *in vivo* metastasis assays using MGC-803 cells infected with QKI5 or control lentivirus and then injected into the lateral tail veins of nude mice. These mice were sacrificed five weeks after injection, and the liver and lung were dissected for microscopic histology (Figure 3E). The number of liver metastasis in mice injected with QKI5 lentivirus-transduced MGC-803 cells was significantly lower than that in mice injected with control lentivirus-infected cells (Figure 3E and 3G). Hematoxylin and eosin (H&E) staining was subsequently performed to assess the pathological properties of the liver tissues, which showed more metastatic nodules in control lentivirus-treated mice compared with QKI5-treated mice (Figure 3F). Similar results were observed in the lung tissues (Figure 3G and 3F), although we did not observe significant changes in outward appearance (Figure 3E). Thus, QKI5 regulated tumorigenesis by inhibiting the proliferative and invasive activities of GC cells.

### QKI5 regulates the alternative splicing of macroH2A1 in GC cells

QKI5, QKI6, and QKI7, are protein isoforms generated by alternative splicing from the common QKI pre-mRNA in mouse and human. QKI5 isoform is a nucleus-cytoplasm shuttling protein, but it is found mostly in the nucleus, whereas QKI6 and QKI7 isoforms are exclusively localized to the cytoplasm QKI5 is a conserved signal transduction and activation of RNA (STAR) family protein that plays an essential role during embryonic and postnatal development. Recent work by Novikov, et al. has showed that QKI level was correlated to the expression of macroH2A1.1 in lung cancer [16]. Moreover, the changes in the alternative splicing of macroH2A1 have been reported in a variety of human cancers including breast [23], colorectal [24], lung [25, 26], testis, bladder, ovarian, endometrial and cervical cancers [26]. Therefore, to test whether QKI5 regulates the alternative splicing of macroH2A1 in GC cells, we used HGC-27, which has a relatively lower endogenous QKI5 level, to restore QKI5 by pcDNA-QKI5 transfection, and SGC-7901, which has a higher endogenous QKI5 level, to deplete QKI5 by two shRNAs specific to QKI5 (Figure 4A). Immunoblotting was performed to confirm the restoration or depletion of QKI5 from the cells (Figure 4A). The changes in QKI5 protein levels led to significant changes in macroH2A1 splicing (Figure 4B). In HGC-27 cells, QKI5 overexpression led to a significant increase in macroH2A1.1 mRNA and a slightly decrease in macroH2A1.2 mRNA levels, whereas total macroH2A1 transcript levels were not significantly altered (Figure 4B). In SGC-7901 cells, we detected a dramatic reduction in macroH2A1.1 mRNA levels in QKI5 knockdown cells compared with the levels in controls. Accordingly, the macroH2A1.2 mRNA level increased upon shRNA treatment (Figure 4B). Notably, the changes in macroH2A1 pre-mRNA alternative splicing observed upon the changes in QKI5 were also apparent when examined at the protein level (Figure 4C). Thus, our data suggested that QKI5 could control the alternative splicing of macroH2A1 in GC cells.

**Figure 4:** QKI5 regulates macroH2A1 alternative splicing in GC cells **A.** QKI5 levels were detected in HGC-27 cells after treatment with pcDNA-QKI5 or pcDNA empty vector, and in SGC-7901 cells after treatment with si-QKI5s or siRNA controls by immunoblotting; **B.** Relative expression of macroH2A1.1, macroH2A1.2, and total macroH2A1 in QKI overexpressing and knockdown cells as described in A; **C.** Immunoblotting of the protein levels of macroH2A1.1, macroH2A1.2, and total macroH2A1 in QKI overexpressing and knockdown cells as described in A; **D.** Expression level of macroH2A1.1 mRNA was detected in 100 pairs of GC tissues and adjacent normal regions by RT-qPCR. **E.** The normalized relative expression of QKI5, mH2A1.1 and mH2A1.2 from the 100 pairs of gastric cancer samples were plotted in a radar graph on a logarithmic scale. **F.** Statistical analysis of the survival probability of macroH2A1.1 high- (n = 10) and low-expressing (n = 50) GC patients using Kaplan–Meier analysis. Statistical analysis is described in the Materials and Methods.

Consistent with the downregulation of QKI5 in GC, the macroH2A1.1 level was significantly reduced in the same 100 pairs of clinic GC tissue and matched adjacent normal tissue samples (Figure 4D). However, the macroH2A1.2 level was negatively correlated with both QKI5 and macroH1A1.1 levels (Figure 4E). Additionally, low macroH1A1.1 level was also associated with poor survival of GC patients (Figure 4F and Supplementary Table 2). These data indicated that QKI5 might suppress GC progression, at least in part, through regulating the production of macroH2A1.1.

### MacroH2A1.1 functions as a tumor suppressor in GC

Based on the above findings, macroH2A1.1 may also play a suppressive role in gastric carcinogenesis. To test this idea, HGC-27 was selected to study the function of macroH2A1.1. Immunoblotting was used to measure the level of macroH2A1.1 protein after transfection of the contrast pcDNA-mH2A1.1, and the results showed that the level of macroH2A1.1 was increased to fourfold in HGC-27 cells (Figure 5A). To confirm the specific effects of macroH2A1.1 on gastric carcinogenesis, another contrast expressing the isoform macroH2A1.2 was used as a control (Figure 5A).

**Figure 5:** Functional analysis of macroH2A1.1 in GC cells **A.** MacroH2A1.1 levels were detected in HGC-27 cells after treatment with pcDNA-macroH2A1.1 or pcDNA empty vector by immunoblotting; **B.** Cell proliferation assay of HGC-27 cells after treatment with pcDNA-macroH2A1.1 or pcDNA using CCK-8; **C.** Flow cytometry was conducted to examine the apoptosis of HGC-27 cells after treatment with pcDNA-macroH2A1.1 or pcDNA and stained with apoptosis markers (FITC-Annexin V and PI). In the apoptosis map, FITC-Annexin V+/PI+ indicates late apoptosis, FITC-Annexin V+/PI− indicates early apoptosis, and FITC-Annexin V−/PI− indicates normal live cells. **D.** Wound healing assays of HGC-27 cells after treatment with pcDNA-macroH2A1.1 or pcDNA. The relative ratio of wound closure per field is shown in the right; **E.** Transwell analysis of HGC-27 cells after treatment with pcDNA-macroH2A1.1 or pcDNA. The relative ratio of invasive cells per field is shown in the right. For all qPCR results, the data are presented as the mean ± SEM, and the error bars represent the standard deviation obtained from three independent experiments. * *p* < 0.05; ** *p* < 0.01. **F.** Pathology analysis of tumor sections from GC tissues and adjacent normal tissues. Immunohistochemistry, H&E staining, and labeling with QKI5 and mH2A1.1 was performed. Bars: 20 μm. * *p* < 0.05; ** *p* < 0.01. The relative ratio of expression is shown in the right.

The CCK-8 proliferation assay in HGC-27 cells indicated that cell growth was suppressed after transfection with pcDNA-mH2A1.1 but not with pcDNA-mH2A1.2 (Figure 5B). Ectopic macroH2A1.1 expression also decreased the early and late apoptosis of HGC-27 cells compared with the control group (Figure 5C). Wound healing assay showed that cell migration was inhibited in pcDNA-mH2A1.1-transfected HGC-27 cells (Figure 5D). To detect whether macroH2A1.1 can inhibit cell invasion ability, transwell invasion assay was performed. As expected, a significant reduction in cell invasiveness was found after macroH2A1.1 overexpression in HGC-27 cells (Figure 5E). As in the CCK-8 assay, the increased macroH2A1.2 had no effects on HGC-27 cell apoptosis, migration, and invasion.

We next investigated whether macroH2A1.1 is expressed at a low level in GC tissues with downregulated QKI5. As expected, immunohistochemistry revealed that macroH2A1.1 staining was significantly decreased in GC tissues (Figure 5F). All these findings indicated that the tumor suppressor role was specific to macroH2A1.1 in GC cells, which was consistent with its alternative splicing regulator QKI5.

### MacroH2A1.1 inhibits the expression of CCNL1 in GC cells

In general, macroH2A1.1 is associated with repressive heterochromatin, in which it colocalizes with other heterochromatin markers, such as histone H3 lysine 27 trimethylation (H3K27me3) [27, 28]. To define macroH2A1.1-regulated genes in GC cells, we compared the existing macroH2A1 ChIP-seq [29, 30] and RNA-seq [31] database and performed qPCR to validate these candidates in HGC-27 cells (Figure 6A). As shown in Figure 6A, CCNL1 displayed the most significant expression changes upon macroH2A1.1 overexpression. Together with its oncogenic roles in several cancers, including, cervical, breast, head and neck cancers [32–34], we selected CCNL1 for further study. Given that a previous study has reported the occupancy of macroH2A1.1 on the genomic locus of the CCNL1 gene, we performed ChIP-PCR analysis and confirmed H2A1.1 occupancy on the upstream of the CCNL1 locus in HGC-27 cells (Figure 6B). Furthermore, increased H2A1.1 binding was observed in HGC-27 cells with overexpressed macroH2A1.1 (Figure 6C). More importantly, the introduction of QKI5 into HGC-27 cells also enhanced H2A1.1 occupancy on the CCNL1 locus (Figure 6C). To understand whether macroH2A1.1 regulates the GC cell phenotype via suppressing CCNL1, we detected the changes in CCNL1 protein expression after macroH2A1.1 overexpression in HGC-27 cells (Figure 6D). Immunoblotting analysis confirmed the decreased protein levels of CCNL1 upon macroH2A1.1 overexpression (Figure 6D). The QKI5-overexpressed HGC-27cells also displayed low CCNL1 expression (Figure 6D).

**Figure 6:** MacroH2A1.1 regulates CCNL1 expression in GC cells **A.** Expression changes in selected target genes were examined by RT-qPCR analyses in HGC-27 cells transfected with pcDNA-macroH2A1.1 or pcDNA. **B** and **C.** Occupancy of macroH2A1 was examined by ChIP-qPCR analyses in untreated HGC-27 cells (B) and in pcDNA-macroH2A1.1- or pcDNA-QKI5-transfected HGC-27 cells (C). #1 and #2 respect the first and second pairs of primers used for PCR analysis. **D.** Immunoblotting of the protein levels of CCNL1 in HGC-27 cells treated with pcDNA-macroH2A1.1, pcDNA-QKI5, or pcDNA. **E.** Expression level of CCNL1 mRNA was detected in 100 pairs of GC tissues and adjacent normal regions by RT-qPCR. **F.** Statistical analysis of survival probability of CCNL1 high- (n = 47) and low-expressing (n = 9) GC patients using Kaplan–Meier analysis. Statistical analysis is described in the Materials and Methods. **G.** Schematic model of the QKI5-macroH2A1.1-CCNL1 cascade in gastric carcinogenesis.

Consistent with the reduced QKI5 and H2A1.1 levels in GC samples, the CCNL1 mRNA level was markedly increased in GC tissues compared with that in normal samples (Figure 6E). High CCNL1 expression was found to be associated with poor survival in GC patients (Figure 6F and Supplementary Table 2). Therefore, the novel QKI5-macroH2A1.1-CCNL1 axis was presented in GC cells (Figure 6G).

## DISCUSSION

GC is the fourth most commonly diagnosed cancer and the second lethal malignancy worldwide; it is the most common gastrointestinal malignancy in East Asia and Eastern Europe [35]. GC is often diagnosed at the advanced stage, accompanied with malignant cell growth and metastasis. In spite of the progress in chemotherapy, radiotherapy, and surgical techniques for GC in recent years, the survival rate of GC patients remains unsatisfactory [36–38]. Although many oncogenes or tumor suppressors have been identified as key regulators in GC tumorigenesis, almost no commonly accepted biomarkers or therapy targets have been established to facilitate the comprehensive management of patients [39, 40]. Therefore, the identification of the novel regulators for GC and a detailed understanding of the molecular mechanisms underlying gastric carcinogenesis will be of great importance to help our understanding of GC. In this study, we demonstrated that the RNA-binding protein QKI5 was significantly downregulated in GC patients and served as a novel regulator of gastric carcinogenesis, suggesting that the restoration of QKI5 expression would provide a new strategy for GC therapy.

QKI which belongs to the STAR family of the KH domain containing RNA-binding proteins, has been found to affect pre-mRNA splicing, mRNA turnover, mRNA translation, and circular RNA formation; QKI has been implicated in different diseases including ataxia, schizophrenia, and tumorigenesis [3, 16, 41, 42]. The QKI-mediated repression of FOXO1 has been shown to contribute to the oncogenesis and progression of breast carcinoma [43, 44]. QKI also impairs self-renewal and tumorigenicity of oral cancer cells via repression of SOX2 [45]. Additionally, QKI suppresses glioblastoma multiforme tumor progression via indirect stabilization of certain miRNAs [46]. Although previous studies have strongly suggested that QKI5 functions as a tumor suppressor in various types of cancer, the identification of its direct functional targets is only beginning. Recent PAR-CLIP crosslinking analyses in human embryonic kidney cells (HEK293T) have indicated that the majority of QKI binding occurs within introns, consistent with its important roles in regulating alternative splicing [47, 48]. For example, Zong et al. reported that QKI5 can inhibit NSCLC cell proliferation and prevent inappropriate activation of the Notch signaling pathway by repressing the inclusion of NUMB alternative exon through competing with a core splicing factor SF1 [3]. They also identified a number of cancer-associated splicing events caused by the downregulation of QKI5. A previous study reported the correlation between QKI level and macroH2A1.1 expression in a variety of cancers, including testicular, lung, bladder, cervical, breast, colon, ovarian, and endometrial cancers [16]. In our study, we established the linkage between QKI5 and macroH2A1.1, an alternative splicing product from macroH2A mRNA, in GC.

MacroH2A1 is one histone variant counterpart that can substitute for at least one copy of H2A in a subset of nucleosomes in vertebrates. The macrodomain of macroH2A may play a role in the modulation of gene expression outcomes via physical interactions with effector proteins, such as PELP1 and PARP1 [27]. MacroH2A1.1 and macroH2A1.2 are splice variants of the same macroH2A1 gene, and each of them bears a unique exon. Similar to most macrodomains, macroH2A1.1's macrodomain can interact with NAD^+^-derived ligands, such as PAR, whereas the macrodomain of macroH2A1.2 cannot. This distinction is functionally important in cancer, in which reduction in macroH2A1.1 occurs in several tumor types and the alteration in macroH2A1.1 expression has important effects on both the proliferation and metastatic potential of cancer cells [18, 28]. In the present study, we demonstrated that macroH2A1.1 inhibited GC cell proliferation, migration, and invasion by repressing CCNL1 expression. Moreover, the reduced macroH2A1.1 in GC cells was due to the downregulated QKI5, so the QKI5-macroH2A1.1-CCNL1 axis might have essential roles in gastric carcinogenesis. The findings of this study have significant implications regarding the understanding of GC pathogenesis. The pleiotropic effects of QKI5 on GC tumorigenesis suggest that QKI5 could be an effective target for antineoplastic therapies.

## MATERIALS AND METHODS

### Clinical specimens and cell lines

GCs and their morphologically normal tissues (located > 3cm away from the tumor) were obtained between November 2011 and May 2015 from 100 GC patients undergoing surgery at the Cancer Hospital of Chinese Academy of Medical Sciences. Tissue samples were cut into two parts. One part was fixed with 10% formalin for histopathological diagnosis, and the other was immediately snap frozen in liquid nitrogen and stored in liquid nitrogen until RNA extraction. The patient characteristics are provided in Supplementary Table 1. The 293T and GC cell line, AGS, HGC-27, MGC-803, BGC-823, SGC-7901 and MKN-45 cell lines were obtained from the American Type Culture Collection and grown in DMEM with 10% FBS (Hyclone) at 37°C in a 5% CO_2_ cell culture incubator.

### Tissue RNA isolation and RT-qPCR

Total RNA was extracted from cells and tissues using Trizol reagent (Invitrogen, CA, USA) according to the manufacturer's instructions. RT-qPCR was conducted to detect the level of RNA transcripts. In brief, cDNA was synthesized by M-MLV reverse transcriptase (Invitrogen) from 5 μg of total RNA. Oligo (dT18) RT primer was used for the reverse transcription of mRNA. RT-qPCR was performed on the Bio-rad CFX96 real-time PCR system (Bio-rad, Foster City, CA, USA) using KAPA PROBE FAST qPCR kits (Kapa Biosystems, MA, USA) and TaqMan probes (Invitrogen) with the following cycling conditions: 95°C for 10 min (initial denaturation), followed by 40 cycles of 95°C for 15 s, 60°C for 60 s. Primers sequences are listed in Supplementary Table 3. GAPDH was used for mRNA normalization.

### Oligonucleotides and constructs

Two siRNAs (specifically for QKI5, si-QKI5-1, and si-QKI5-2) and control siRNAs (Si-control) were synthesized by Dharmacon and transfected (100 nM) using DharmFECT1. For QKI5 overexpression, the human QKI5 (NM_006775) cDNA ORF was inserted into the pcDNA vector (pcDNA-QKI5) downstream of the CMV promoter. For macroH2A1.1 and macroH2A1.2 overexpression, the human macroH2A1.1 and macroH2A1.2 cDNA ORF was inserted into the pcDNA vector downstream of the CMV promoter (pcDNA-mH2A1.1 and pcDNA-mH2A1.2), respectively. Transfection of these constructs was carried out with either Lipofectamine 2000 (Invitrogen, Carlsbad, CA, USA) for 293T cells or Lipofectamine™ LTX & PLUS for HGC-27 and MGC-803 according to the manufacturer's protocols.

### Cell proliferation assay

HGC-27 and MGC-803 cells were incubated in 10% CCK-8 (DOJINDO, Japan) diluted in normal culture medium at 37°C until visual color conversion occurred. Proliferation rates were determined at 0, 24, 48, 72 and 96 h after transfection. The absorbance of each well was measured with a microplate reader set at 450 and 630 nm. All experiments were performed in triplicate.

### Cell apoptosis assay

To detect the apoptosis of HGC-27 and MGC-803 cells, flow cytometric analysis was conducted with an Annexin V-FITC/PI Apoptosis Detection Kit (KeyGEN Biotech, Nanjing, China) according to the manufacturer's instructions. Data acquisition and analysis were performed using MoFlow (Beckman Coulter, Atlanta, GA, USA).

### Cell migration and invasion assays

HGC-27 and MGC-803 cells were grown to confluence on 12-well plastic dishes and treated with siRNAs or control. At 24 h after transfection, linear scratch wounds (in triplicate) were created on the confluent cell monolayers using a 200 μL pipette tip. To remove cells from the cell cycle prior to wounding, cells were maintained in serum-free medium. To visualize migrated cells and wound healing, images were obtained at 0, 24, and 48 h. Ten areas were selected randomly from each well, and the cells in three wells of each group were quantified.

For the invasion assays, after 24 h of transfection, 1 × 10^5^ HGC-27 or MGC-803 cells in serum-free media were seeded onto the transwell migration chambers (8 μm pore size; Millipore, Switzerland), in which the upper chamber of an insert was coated with Matrigel (Sigma-Aldrich, USA). Media containing 20% FBS were added to the lower chamber. After 24 h, the non-invading cells were removed with cotton wool. Invasive cells located on the lower surface of the chamber were stained with May-Grunwald-Giemsa stain (Sigma-Aldrich, USA) and counted using a microscope (Olympus, Tokyo, Japan). Experiments were independently repeated three times.

### Chromatin immunoprecipitation (ChIP) assay

Anti-mH2A1.1 antibody (Cell Signaling, 12455) and rabbit isotype control IgG (Abcam, ab27472) were used for ChIP studies. HGC-27 cells were collected and cross-linked with 1% formaldehyde for 10 min, washed in cold PBS buffer, resuspended in lysis buffer (0.1% SDS, 0.5% Triton X-100, 20 mM Tris-HCl [pH 8.1], 150 mM NaCl, protease inhibitor, Roche), and sonicated to obtain chromatin fragments between 200 bp and 1000 bp. Sonicated chromatin was resuspended in IP buffer and incubated overnight at 4°C with magnetic bead-conjugated antibodies (Santa Cruz Biotechnologies). The IP was then washed with lysis buffer, LiCl buffer (0.25 M LiCl, 1% NP-40, 1% deoxycholate, 1 mM EDTA and 10 mM Tris-HCl [pH 8.1]) and TE buffer and then eluted in elution buffer (1% SDS, 0.1 M NaHCO_3_). DNA was then recovered by reversing the crosslinks and purified using a QIAGEN purification kit. An unenriched sample of DNA was treated in a similar manner to serve as the input. The primers used for the ChIP-PCR experiment are listed in Supplementary Table 3.

### Western blot analysis

Immunoblotting analysis was carried out using standard methods. Proteins were separated by 10% SDS-PAGE and transferred onto PVDF membranes (Millipore Corporation, Billerica, MA, USA). Membranes were blocked overnight with 5% non-fat dried milk for 2 h and incubated with anti-QKI5 antibody (Millipore, AB9904) at 1:2000 dilution; anti-mH2A1.1 antibody (Cell Signaling, 12455) at 1:500 dilution; anti-mH2A1.2 antibody (Cell Signaling, 4827) at 1:500 dilution; and anti-GAPDH antibody (Proteintech) at 1:50,000 dilution overnight at 4°C. After washing with TBST (10 mM Tris, pH 8.0, 150 mM NaCl, and 0.1% Tween 20), the membranes were incubated for 2 h at room temperature with goat anti-rabbit antibody (Zsgb-bio, Beijing, China) at 1:20,000.

### Immunohistochemistry and scoring

Paraffin-embedded sections of tissues obtained from the GC patients were cut into coated slides, deparaffinized with xylol, and rehydrated through 90%, 80% and 70% ethanol. After washing in water, the slides were autoclaved for 3 min at 1.5 atm in sodium citrate buffer for antigen retrieval. Endogenous peroxidase activity was blocked with hydrogen peroxidase for 5 min at room temperature. The sections were incubated with diluted antibodies (QKI5, 1:250; mH2A1.1, 1:80) for 30 min, and subsequently washed with 1 × TBS and incubated with secondary antibody for another 30 min. Diaminobenzidine (DAB) and the hematoxylin chromogen (Dako, Glostrup, Denmark) method was used. The sections were subsequently examined by light microscopy, and the staining intensity was determined. The IHC results (Q) are scored by multiplying the percentage of positive cells (P) by the intensity (I). Then, the relative scores of GC samples are normalized to the control.

### Tumorigenicity and tumor metastasis formation assay *in vivo*

All experimental procedures involving animals were performed in accordance with the Guide for the Care and Use of Laboratory Animals (NIH publications Nos. 80–23, revised 1996) and according to the institutional ethical guidelines for animal experiments. Lenti-GFP (Control) and Lenti-QKI5 (QKI5)-transduced MGC-803 cells (1 × 10^7^) were suspended in 100 μL of PBS and then injected subcutaneously into either side of the posterior flank of the same female BALB/c athymic nude mouse at five-six weeks of age. Five nude mice were included in each group and tumor growth was examined every three days over a course of four weeks. Tumor volume (V) was monitored by measuring the length (L) and width (W) of the tumor with calipers, and it was calculated with the formula V = (L × W2) × 0.5.

We also used the nude mice xenograft model to estimate the metastatic ability of the control- and QKI5-transduced MGC-803 cells *in vivo*. Viable cells (5 × 10^5^) were resuspended in 0.1 mL of PBS and injected into the lateral tail vein. Five weeks after the injection, we monitored tumor metastases using a live animal bioluminescence imaging system. Mice were then killed and the lungs and livers were extracted and fixed in 4% paraformaldehyde in PBS. Paraffin embedding, sectioning and staining with H&E were performed. Visible lung and liver metastases were measured and counted using a microscope.

### Statistics

Each experiment was repeated at least three times. Student's t-test (two-tailed) was performed and three-group data were analyzed using one-way ANOVA. All statistical analyses were performed using SPSS 16.0 software (SPSS Inc., Chicago, IL, USA). Statistically significance was set at *P* < 0.05.

## SUPPLEMENTARY TABLES


